RETRACTED

# Protective Effects of Celastrol on Diabetic Liver Injury via TLR4/MyD88/NF-*κ*B Signaling Pathway in Type 2 Diabetic Rats

**DOI:** 10.1155/2016/2641248

**Published:** 2016-01-19

**Authors:** Li-ping Han, Chun-jun Li, Bei Sun, Yun Xie, Yue Guan, Ze-jun Ma, Li-ming Chen

**Affiliations:** 2011 Collaborative Innovation Center of Tianjin for Medical Epigenetics, Key Laboratory of Hormone and Development, Ministry of Health, Metabolic Disease Hospital and Tianjin Institute of Endocrinology, Tianjin Medical University, Tianjin 300070, China

## Abstract

Immune and inflammatory pathways play a central role in the pathogenesis of diabetic liver injury. Celastrol is a potent immunosuppressive and anti-inflammatory agent. So far, there is no evidence regarding the mechanism of innate immune alterations of celastrol on diabetic liver injury in type 2 diabetic animal models. The present study was aimed at investigating protective effects of celastrol on the liver injury in diabetic rats and at elucidating the possible involved mechanisms. We analyzed the liver histopathological and biochemical changes and the expressions of TLR4 mediated signaling pathway. Compared to the normal control group, diabetic rats were found to have obvious steatohepatitis and proinflammatory cytokine activities were significantly upregulated. Celastrol-treated diabetic rats show reduced hepatic inflammation and macrophages infiltration. The expressions of TLR4, MyD88, NF-*κ*B, and downstream inflammatory factors IL-1*β* and TNF*α* in the hepatic tissue of treated rats were downregulated in a dose-dependent manner. We firstly found that celastrol treatment could delay the progression of diabetic liver disease in type 2 diabetic rats via inhibition of TLR4/MyD88/NF-*κ*B signaling cascade pathways and its downstream inflammatory effectors.

## 1. Introduction

Diabetic liver damage was mainly caused by fatty infiltration of the liver leading to nonalcoholic fatty liver disease (NAFLD). NAFLD is the hepatic manifestation of the metabolic syndrome and covers a disease spectrum ranging from simple steatosis with no inflammation to steatosis with varying degrees of inflammation (steatohepatitis, NASH) to fibrosis, cirrhosis, and hepatocellular carcinoma [1, 2]. Among them, NASH is an important turning point and the complex cellular components of the innate immune system play an essential role in perpetuating and modulating the inflammatory response in the liver [3].

The Toll-like receptors (TLRs) family is one of the best-characterized pattern recognition receptor families and is responsible for sensing invading pathogens outside of the cell [4, 5]. Once a molecular pattern has been recognized by the TLRs, downstream signaling is initiated, resulting in the innate immune and inflammatory responses. TLR4 is one of the receptors which is related to whole-body, low-grade chronic inflammatory diseases [6] and contributes to macrophage infiltration in experimental models of diabetes-related liver injury [7]. NF-*κ*B is a ubiquitous and well-known transcription factor responsible for the rapid induction of many cytokines implicated in the immune and inflammation [8]. There is evidence showing that NF-*κ*B is activated in NASH and liver fibrosis models in vivo and in vitro [9, 10]. Moreover, the TLR4 signaling pathway can activate NF-*κ*B and induce the expression of proinflammatory genes [11]. Therefore, downregulation of the expression of TLR4/NF-*κ*B signaling pathways and its downstream inflammatory effectors might represent a novel treatment strategy for reducing diabetic liver injury.

RETRACTED

Celastrol (C_29_H_38_O_4_) is a pharmacologically active pentacyclic-triterpene extract from the roots of traditional Chinese herbal plant* Tripterygium wilfordii* Hook.f. (TwHF, thunder god vine). Recent research reported that celastrol had potent anti-inflammatory and immunosuppressive properties. To date, celastrol has been widely used for the treatment of various diseases, such as cancer, neurodegenerative disease, and autoimmune diseases [12–15]. The latest research reported that celastrol was able to effectively alleviate high-fat mediated cardiovascular disease and diabetic nephropathy [16, 17]. But there is still a lack of data describing the anti-inflammatory and immunosuppressive activities of celastrol on diabetic liver injury. The present study was conducted using rat model of T_2_DM induced by high-fat diet combined with low-dose STZ to investigate the effects of celastrol on hepatic tissues and explore its possible mechanisms.

## 2. Materials and Methods

### 2.1. Animals

This study was carried out in strict accordance with the recommendations in the Guide for the Care and Use of Laboratory Animals of the National Institutes of Health. The protocol was approved by the Animal Care and Use Committee on the Ethics of Animal Experiments of Tianjin Medical University (Tianjin, China). All steps were taken to avoid animal suffering at each stage of the experiment. Seventy-five healthy male Sprague-Dawley rats, 4~5 weeks of age, weighing 161 ± 9 g, were purchased from Beijing HFK Technology Co., Ltd. (Beijing, China). All of the rats were housed under pathogen-free conditions and were provided with rat chow and water ad libitum. The animals were maintained at a controlled temperature (22°C ± 2°C), humidity (55% ± 10%), and photoperiod (12 h light/dark cycles). The animals were acclimatized to the laboratory for 1 week before the experiments. 15 rats were randomly selected as normal control group (NC group) and fed with a conventional diet. The remaining 60 rats were given high-fat diet (formula is sucrose 10%, lard 10%, cholesterol 1%, and sodium cholate 0.3%, and the rest is composed of the basic diet, irradiated by cobalt-60, provided by HFK Technology Co., Ltd., Beijing, China). After 8 weeks of feeding, fasting plasma glucose (FPG) and insulin (FINS, Radioimmunoassay), and triglycerides, total cholesterol levels were measured, and HOMA-IR and HOMA-*β* were assessed by homeostasis model (HOMA-IR = FPG × FINS/22.5, HOMA-*β* = 20 × FINS/(FPG − 3.5)). When insulin resistance occurred, STZ 30 mg/kg (pH 4.32) intravenously was injected to induce rat model of T_2_DM. 15 normal rats were intravenously injected with sodium citrate buffer. The tail blood glucose was measured, which is greater than 16.7 mmol/L to be thought successful. The diabetic rats were randomly assigned to four groups: rats receiving vehicle only (DM group) and three groups of rats receiving different doses of celastrol.

RETRACTED

### 2.2. Celastrol Solution

Purified celastrol was purchased from Sigma Chemical Co. (Sigma, St. Louis, MO, USA) and stored at −20°C. Celastrol was freshly dissolved in 10% dimethyl sulfoxide (DMSO) before use in the experiments, and vehicle (distilled water containing 10% DMSO) was used as a control. Treatment rats were administered by oral gavage with low-dose celastrol (100 *μ*g/kg, CL group), medium-dose celastrol (200 *μ*g/kg, CM group), and high-dose celastrol (500 *μ*g/kg, CH group) once daily for 8 weeks.

### 2.3. Biochemical Analysis

Rats were sacrificed under anesthesia by i.p. injection of sodium pentobarbital. We measured liver weight and calculated liver index (liver weight/body weight). After centrifugation of the blood samples, the serum concentrations of glucose, alanine aminotransferase, aspartate aminotransferase, blood urea nitrogen, creatinine, total cholesterol, triglyceride, and high density lipoprotein cholesterol were measured using an automatic clinical analyzer (7600A-020, HITACHI Ltd., Tokyo, Japan). Serum IL-1*β* and TNF*α* levels were measured using an enzyme-linked immunosorbent assay (ELISA) kit (Cusabio Biotech, USA). Liver tissue was analyzed for total cholesterol and triglyceride contents (Jiancheng Bioengineering Institute, Nanjing, China), according to the manufacturer's instructions.

### 2.4. Histopathological Evaluations

Sections from the livers were removed and fixed in 10% neutral-buffered formalin and embedded in paraffin and stained with hematoxylin-eosin and Masson's trichrome (MT) for histological analysis.

RETRACTED

### 2.5. Immunohistochemistry Staining

The sectioned slides were stained according to standard protocols described previously. Paraffin-embedded sections of hepatic tissue were deparaffinized, dehydrated, and stained immunohistochemically for detection of mouse monoclonal anti-CD68 antibody (diluted 1 : 200 in PBS; Abcam, UK), mouse monoclonal anti-TLR4 antibody (diluted 1 : 100 in PBS; Abcam, UK), rabbit polyclonal anti-MyD88 antibody (diluted 1 : 100 in PBS; Bioworld technology, Co. Ltd., Nanjing, China), rabbit polyclonal anti-NF-*κ*Bp65 antibody (diluted 1 : 1000 in PBS; Abcam, UK), rabbit polyclonal anti-IL-1*β* antibody (diluted 1 : 100 in PBS; Abcam, UK), and rabbit polyclonal anti-TNF*α* antibody (diluted 1 : 100 in PBS; Abcam, UK) by sequential incubation. A peroxidase-linked secondary antibody and diaminobenzidine (Sungene Biotech Co., Ltd., Tianjin, China) were used to detect specific immunostaining. The slides were rinsed twice and counterstained with hematoxylin. As negative controls for nonspecific binding of the secondary antibody, sections from the same samples were processed without the primary antibody.

### 2.6. Real-Time Reverse Transcription Polymerase Chain Reaction (RT-PCR)

All primers were synthesized by AuGCT Biotechnology (Beijing, China). The primer for rat glyceraldehyde-3-phosphate dehydrogenase gene was used as housekeeping gene. The real-time PCR primer sequences used for PCR were shown in Table 1. Total RNA was isolated from the liver sections with TRIzol reagent (Invitrogen Life Technologies, Carlsbad, CA, USA). cDNA synthesis was performed using the High-Capacity cDNA Reverse Transcription kit (Applied Biosystems, Foster City, CA, USA) according to the manufacturer's instructions. Real-time PCR was performed in 10 *μ*L that contained 5 *μ*L of 2×SYBR Green Premix Ex TaqTM (Takara Biotechnology, Japan), 1 *μ*L of cDNA, 3 *μ*L of distilled water, and 0.5 *μ*L of each primer. PCR was carried out in a thermal cycler (Bio-Rad, Hercules, CA, USA). Initial denaturation was carried out at 95°C for 3 min, followed by 45 cycles of denaturation for 10 s at 95°C, annealing for 30 s at the appropriate temperature, and extension for 20 s at 72°C. The mRNA levels were normalized against the mRNA levels of the housekeeping gene GAPDH. Gene expression and data analysis were monitored using the CFX Manager Software (version 1.6, Bio-Rad, CA, USA). Relative quantification was performed using the 2^−ΔΔCt^ method which results in ratios between target genes and a housekeeping reference gene.

### 2.7. Western Blotting Analysis

Proteins were extracted using RIPA buffer (Thermo, USA), according to the manufacturer's instructions, and the protein concentrations were measured using a BCA protein assay kit (Thermo, USA). An equal amount of protein from each sample was subjected to sodium dodecyl sulfate- (SDS-) polyacrylamide gel electrophoresis and then transferred to polyvinylidene difluoride (PVDF) membranes (Millipore, USA). Membranes were blocked with 5% milk for 2 h at room temperature and incubated overnight at 4°C with primary antibodies, including TLR4 (1 : 1000), MyD88 (1 : 1000), NF-*κ*Bp65 (1 : 1000), phospho-I*κ*B*α* (p-I*κ*B*α*, 1 : 500), IL-1*β* (1 : 1000), TNF*α* (1 : 1000), and internal control *β*-actin (1 : 10000, Sungene Biotech Co., Ltd., Tianjin, China). Membranes were washed twice for 10 min in 1×TBST and then incubated with HRP-conjugated secondary antibodies (goat anti-rabbit IgG: 1 : 12500; goat anti-mouse IgG: 1 : 12500, Sungene Biotech Co., Ltd., Tianjin, China) for 2 h. Membranes were then washed twice for 10 min in 1×TBST. Proteins were visualized by ECL (Millipore, USA), and blots were scanned in dark room. Densitometry analysis of bands was performed with the Image J software.

RETRACTED

### 2.8. Statistical Analysis

Statistical analysis was performed by using SPSS 17.0 version (IBM SPSS Statistics, IBM Corporation, Armonk, NY, USA) and GraphPad Prism 5.0 software (GraphPad Software, Inc., La Jolla, Calif, USA). Quantitative data were expressed as mean ± standard error of the mean (SEM). The significance of the data obtained was evaluated using the one-way analysis of variance (*one-way ANOVA*), followed by* LSD*-test. A value of *P* < 0.05 was considered statistically significant.

## 3. Results

### 3.1. Parameters after 8-Week High-Fat Feeding

Compared with the NC group, total cholesterol and triglycerides levels and the indexes of HOMA-IR and HOMA-*β* of high-fat rats were significantly higher, but there were no changes for blood glucose. These results showed that insulin resistance occurred after 8-week high-fat feeding (Table 2).

### 3.2. Effects of Celastrol on Physical and Biochemical Parameters in Rats

Physical and biochemical parameters for the different groups of rats are shown in Table 3. Compared with the NC group, the body weights of diabetic rats were significantly lower, and blood glucose, serum and liver TC, TG levels, and liver index were significantly higher. Rats given celastrol had no changes in blood glucose, serum lipid, and body weights but showed lower liver TC, TG contents, and liver index in the CH group. No significant differences were observed for ALT, AST, BUN, and SCr levels in all groups of rats.

### 3.3. Effects of Celastrol on Histological Changes of Hepatic Tissues in Rats

As shown in H&E staining sections in Figure 1(a), there was clear structure of hepatic lobule, and hepatocytes radially arranged around the central vein, no obvious inflammatory cell infiltration and Kupffer cells proliferation in the NC group. Hepatic lobular structure generally disappeared, and diffuse large bubble-like hepatocyte steatosis and ballooning with obvious inflammatory cell infiltration around portal area were observed in the DM group. Lesions in treatment group were less than that in the DM group, particularly in the CH group. Masson's trichrome staining (Figure 1(b)) showed weak coloration which appeared along the vascular wall of the portal vein and portal area in the NC group. However, diabetic rats showed more fibrosis changes around perisinusoidal spaces and the portal area. The degree of fibrosis observed in hepatic tissues was much lower in celastrol-treated rats than diabetic rats. As a macrophage-specific marker, CD68 staining showed that there was more Kupffer cells infiltration in diabetic rats than in the NC rats. Celastrol administration decreased CD68 expression, particularly in the CH group (Figure 1(c)).

RETRACTED

### 3.4. Effects of Celastrol on Expressions of TLR4 and Downstream Signaling Ligand MyD88 of Hepatic Tissues in Rats

TLR4 expression was observed only in a few hepatocytes in the NC group with immunohistochemical staining. In contrast, higher expression of TLR4 was observed in the cytoplasm and membranes of hepatocytes and Kupffer cells in the DM group and lower expression in celastrol treatment group, especially in the CH group. Similar patterns of expression were observed for MyD88 in the cytoplasm (Figures 2(a) and 2(b)). RT-PCR and Western Blotting analysis showed that TLR4, MyD88 mRNA, and protein levels in the hepatic tissues of the DM group were significantly increased compared with those of the NC group. Additionally, levels of all transcripts and expressions were decreased in rats in celastrol treatment groups. Moreover, celastrol administration decreased expressions in a dose-dependent manner (Figures 2(c)–2(f)).

### 3.5. Effects of Celastrol on Expressions of NF-*κ*B and p-I*κ*B*α* of Hepatic Tissues in Rats

NF-*κ*B staining was observed with immunohistochemical staining only in a few hepatocytes in the NC group. In contrast, higher expression was observed in the nucleus in the DM group and lower expression in celastrol treatment group, especially in the CH group. RT-PCR and Western Blotting showed that NF-*κ*Bp65 and p-I*κ*B*α* expressions in the DM group were significantly increased compared with those in the NC group. Additionally, expressions were decreased in celastrol treatment groups in a dose-dependent manner (Figures 3(a)–3(d)).

RETRACTED

### 3.6. Effects of Celastrol on Expressions of Downstream Inflammatory Cytokines IL-1*β* and TNF*α* of Hepatic Tissues and Serum in Rats

IL-1*β* and TNF*α* staining were observed in the cytoplasm. Compared with the NC rats, there were more positive expressions in diabetic rats, all with reduced staining observed in rats treated with different doses of celastrol, especially in the CH group (Figures 4(a) and 4(b)). Similar to immunohistochemical staining, IL-1*β*, TNF*α* mRNA, and protein levels in the hepatic tissues and serum contents in the DM group were significantly increased compared with those in the NC group and were decreased in celastrol administration rats in a dose-dependent manner (Figures 4(c)–4(h)).

## 4. Discussion

Diabetes mellitus often coexists with different metabolic-related syndromes, such as dyslipidemia, hypertension, and NAFLD [7]. In our present study, experimental type 2 diabetes' rat model was induced by 8-week high-fat feeding combined with low-dose STZ injection [18]. Therefore, our experimental diabetic model is very similar to the pathogenesis of type 2 diabetes. Our observation documented that diabetic rats showed increased glucose combined with insulin resistance and abnormal lipid profiles, liver pathological changes including obvious inflammation and fibrosis, and more macrophage infiltration compared with normal rats, in line with steatohepatitis changes. But serum ALT and AST levels were not obviously increased, because of relative early stage of NAFLD. The earlier stage of NASH may only show mild pathological changes and may not result in the elevated liver enzymes. The latest research demonstrated that celastrol (100 *μ*g–1 mg/kg) was able to effectively suppress weight and improve lipid accumulation in organs including the kidney, liver, and adipose tissue in db/db mice [17, 19]. In our study, we applied relative low three dosages of celastrol (100 *μ*g/kg, 200 *μ*g/kg, and 500 *μ*g/kg) according to previous literature [17, 19]. After 8 weeks of administration, although there were no significant differences in serum glucose, triglycerides, and total cholesterol levels compared with the nontreatment group, the levels of triglycerides and total cholesterol of hepatic tissue were significantly decreased and the liver pathological changes were differently lessened in the treatment groups in a dose-dependent manner. The results showed that early use of celastrol could improve lipid metabolism disorders in liver and delay the progression of diabetic fatty liver disease.

TLR4 signaling pathway is more common pathway factor and has an important regulatory role in stimulating the immune and inflammatory response-related genes expression in the liver, which is activated by accumulation of fatty acids of the liver, particularly saturated fatty acids [3, 20]. Csak et al. found that inactivation of TLR4 in methionine-/choline-deficient mice resulted in a marked attenuation of steatohepatitis induced by a diet [21]. Consequently, targeting TLR4 provides a promising intervention strategy for the prevention or treatment of diabetic fatty liver disease [3]. T_2_DM displays insulin resistance, abnormal glucose and lipid, oxidative stress, and so forth, leading to an increase of endogenous and exogenous ligands of TLR4 such as FFAs, LPS, and endotoxin, and activates TLR4 signaling pathway to induce liver injury [22], in line with our results. As mentioned above, we found that TLR4 were expressed generally on hepatocytes and Kupffer cells in diabetic liver and the consistent upregulation with immunohistochemical staining, RT-PCR, and Western Blotting, and the treatment with celastrol significantly reduced the expressions of TLR4. Similar results were also shown in Kim's research [17].

RETRACTED

TLR4 is initiated through two different pathways, the MyD88-dependent pathway and the MyD88-independent pathway [3]. MyD88 is a critical downstream signaling ligand of TLR4 receptor complex and also is an important adapter protein of NF-*κ*B signaling pathway, contributing to the expression of inflammatory genes. Spruss et al. showed that a significant increase of MyD88 mRNA in high-fat- and fructose-induced hepatic steatosis but inactivation of TLR4 led to a significant decrease in MyD88 mRNA level [23]. Miura et al. proved that the absence of MyD88 prevented hepatic steatosis [24]. Therefore, MyD88 served as the key TLR4 adaptor protein, linking the receptors to downstream kinases in fatty liver disease. Our study showed that TLR4 and MyD88 gene and protein expressions were consistently increased in diabetic rat liver and suppressed with celastrol administration, indicating that anti-inflammatory effect of celastrol might be through TLR4/MyD88-dependent signal transduction pathway.

NF-*κ*B activation is essential for hepatic inflammatory recruitment in steatohepatitis, uniformly found in human NASH and animal models [25–27]. NF-*κ*Bp65 subunit binds to its inhibitory counterpart I*κ*B*α* and other I*κ*B proteins to form P65-I*κ*B trimer which is located in the cytoplasm as an inactive complex. Following I*κ*B*α* phosphorylation and degradation, the activated NF-*κ*Bp65 is disassociated from I*κ*B*α* and shifts to nuclei where it binds to specific DNA motifs to regulate transcriptional activity of its target genes [28]. Therefore, I*κ*B*α* phosphorylation is an indispensable process, which leads to the translocation and activation of NF-*κ*Bp65. In our study we found that hepatocyte NF-*κ*Bp65 was higher expressed in the nuclei in the diabetic rats, along with upregulated p-I*κ*B*α* expressions. But in the celastrol-treated rats, p-I*κ*B*α* and NF-*κ*Bp65 expressions were significantly reduced and NF-*κ*Bp65 was rarely seen in the nuclei. NF-*κ*B was downstream activator of TLR4, involved in TLR4/MyD88-dependent signaling pathway and induced transcriptional expression of multiple proinflammatory chemokines (e.g., TNF*α* and IL-1*β*) associated with liver inflammation [6]. Moreover, proinflammatory chemokines could also upregulate the activity of NF-*κ*B to form a positive feedback regulation mechanism and enhance inflammatory response further [29]. Our study showed that celastrol could inhibit the activation of NF-*κ*B and subsequently suppress signaling cascades that avoid the release of inflammatory response factors TNF*α* and IL-1*β*.

RETRACTED

In the present study, TLR4/MyD88/NF-*κ*B-mediated inflammatory pathways were activated during the progression of diabetic liver disease, resulting in macrophages and other killer cell chemotaxes and aggregation and celastrol could significantly attenuate liver inflammation immune response. But, as a limitation of this study, our approach is only an initial experiment in vivo; further studies will be required in vitro in order to explore its definite mechanisms, which should provide valuable insights into the development of new treatments for diabetic liver injury.

## 5. Conclusion

In summary, our study firstly confirmed that celastrol provided a protective effect against target organ damage in type 2 diabetes rats through inhibition of proinflammatory development in hepatic tissue. These findings suggest that the TLR4/MyD88/NF-*κ*B signaling cascade pathways may be a useful new therapeutic target and celastrol is a promising agent for the pharmacological treatment of diabetic liver injury.

## Figures and Tables

**Figure 1:** Celastrol exhibited protective effects on livers in diabetic rats. (a) H&E staining (×400) showed hepatic steatosis with lobular inflammation and ballooning of hepatocytes in diabetic rats. Alleviation of the infiltration of inflammatory cells and hepatic steatosis were observed in diabetic rats treated with celastrol. (b) Masson's staining (×400) showed mild fibrosis changes around perisinusoidal spaces and the portal area in diabetic rats. The degree of fibrosis decreased in celastrol-treated rats. (c) Immunohistochemistry staining of CD68. More Kupffer cells infiltration was detected in diabetic rats and was downregulated by celastrol administration.

RETRACTED

**Figure 2:** Celastrol administration downregulated the expressions of the TLR4 and MyD88 in diabetic rats liver. (a-b) Immunohistochemical staining of TLR4 and MyD88 (×400). (c-d) Relative mRNA expression levels of TLR4 and MyD88. (e-f) Relative protein expression levels of TLR4 and MyD88 were analyzed by Western Blotting, and the ratio of TLR4/actin and MyD88/actin was shown. The results are expressed as mean ± SEM, ^A^ *P* < 0.05 versus NC group; ^B^ *P* < 0.05 versus DM group; ^C^ *P* < 0.05 versus CL group; ^D^ *P* < 0.05 versus CM group.

**Figure 3:** Celastrol administration downregulated NF-*κ*B and p-I*κ*B*α* expressions in diabetic rats liver. (a) Immunohistochemical staining of NF-*κ*B (×400). (b) Relative mRNA expression levels of NF-*κ*B. (c-d) Relative protein expression levels of p-I*κ*B*α* and NF-*κ*Bp65 were analyzed by Western Blotting, and the ratio of NF-*κ*B/actin and p-I*κ*B*α*/actin was shown. The results are expressed as mean ± SEM, ^A^ *P* < 0.05 versus NC group; ^B^ *P* < 0.05 versus DM group; ^C^ *P* < 0.05 versus CL group; ^D^ *P* < 0.05 versus CM group.

**Figure 4:** Celastrol administration downregulated downstream inflammatory cytokine IL-1*β* and TNF*α* expressions in diabetic rats liver. (a-b) Immunohistochemical staining of IL-1*β* and TNF*α* (×400). (c-d) Relative mRNA expression levels of IL-1*β* and TNF*α*. (e-f) Relative protein expression levels of IL-1*β* and TNF*α* were analyzed by Western Blotting, and the ratio of IL-1*β*/actin and TNF*α*/actin was shown. (g-h) Serum contents of IL-1*β* and TNF*α*. The results are expressed as mean ± SEM, ^A^ *P* < 0.05 versus NC group; ^B^ *P* < 0.05 versus DM group; ^C^ *P* < 0.05 versus CL group; ^D^ *P* < 0.05 versus CM group.

**Table 1:** Sequences of real-time PCR primers.

Primer name	Sequence	Annealing temperature	Size
TLR4	Forward 5′-ATGAGGACTGGGTGAGAAAC-3′	52°C	161 bp
	Reverse 5′-CACCACCACAATAACTTTCC-3′		

MyD88	Forward 5′-TGGTGGTTGTTTCTGACGAT-3′	58.4°C	165 bp
	Reverse 5′-CGCAGATAGTGATGAACCGT-3′		

NF-*κ*B	Forward 5′-AAAAACGCATCCCAAGGTGC-3′	52°C	185 bp
	Reverse 5′-AAGCTCAAGCCACCATACCC-3′		

IL-1*β*	Forward 5′-GGACAGAACATAAGCCAACA-3′	61.4°C	127 bp
	Reverse 5′-CTTTCATCACACAGGACAGG-3′		

TNF*α*	Forward 5′-TCCCAGGTTCTCTTCAAGG-3′	61.4°C	177 bp
	Reverse 5′-GTACATGGGCTCATACCAG-3′		

GAPDH	Forward 5′-GCAAGTTCAACGGCACAG-3′	52°C	218 bp
	Reverse 5′-GCCAGTAGACTCCACGACAT-3′		

PCR: polymerase chain reaction; TLR4: Toll-like receptor 4; MyD88: myeloid differentiation factor 88; NF-*κ*B: nuclear factor-kappa B; IL-1*β*: interleukin-1 beta; TNF*α*: tumor necrosis factor alpha; GAPDH: glyceraldehyde-3-phosphate dehydrogenase.

**Table 2:** Glucose and islet function parameters after 8-week high fat feeding.

Group	FPG (mmol/L)	TG (mmol/L)	TC (mmol/L)	FINS (mIU/L)	HOMA-IR	HOMA-*β*
NC	5.7 ± 0.5	1.3 ± 0.4	2.0 ± 0.2	25.1 ± 4.1	6.5 ± 1.7	230.7 ± 28.7
High-fat	6.1 ± 0.7	3.0 ± 0.7^a^	3.2 ± 0.5^a^	31.6 ± 6.1^a^	8.6 ± 2.3^a^	259.8 ± 42.1^a^

FPG: fasting plasma glucose; TG: triglycerides; TC: total cholesterol; FINS: fasting insulin; IR: insulin resistance. Data are expressed as mean ± SEM, ^a^ *P *< 0.05 versus NC group.

RETRACTED

**Table 3:** Physical and biochemical parameters for rats evaluated in this study.

	NC	DM	DM + CL	DM + CM	DM + CH
Glucose (mmol/L)	6.0 ± 0.2	28.2 ± 3.0^a^	25.3 ± 7.1^a^	26.8 ± 6.1^a^	25.0 ± 4.2^a^
Body weight (g)	442.7 ± 43.8	298.6 ± 37.1^a^	309.4 ± 24.2^a^	303.4 ± 29.5^a^	311.3 ± 30.8^a^
Liver index (g/100 g)	2.67 ± 0.23	4.51 ± 0.35^a^	4.42 ± 0.55^a^	4.27 ± 0.44^a^	3.9 ± 0.27^a,b^
Serum TG (mmol/L)	1.5 ± 1.2	4.4 ± 1.8^a^	4.1 ± 2.1^a^	3.7 ± 2.2^a^	3.5 ± 1.4^a^
Serum TC (mmol/L)	2.2 ± 1.2	6.9 ± 0.9^a^	6.5 ± 2.0^a^	6.4 ± 1.7^a^	6.0 ± 2.1^a^
HDL-C (mmol/L)	0.6 ± 0.1	0.5 ± 0.1	0.5 ± 0.1	0.6 ± 0.1	0.6 ± 0.2
ALT (U/L)	49.7 ± 9.5	55.1 ± 5.1	52.0 ± 9.4	52.7 ± 8.9	50.8 ± 9.1
AST (U/L)	105.1 ± 18.4	109.4 ± 8.4	112.6 ± 9.7	104.3 ± 13.6	104.8 ± 10.5
BUN (mmol/L)	10.9 ± 2.0	10.7 ± 1.6	10.5 ± 1.6	10.9 ± 1.2	9.8 ± 1.8
SCr (*μ*mol/L)	32.8 ± 4.4	31.3 ± 3.3	30.6 ± 3.7	31.4 ± 3.2	30.7 ± 4.1
Liver TG (mg/gprot)	95.8 ± 18.6	412.4 ± 57.8^a^	388.3 ± 38.1^a^	342.4 ± 45.8^a^	228.3 ± 27.5^a,b^
Liver TC (mg/gprot)	40.3 ± 10.1	134.4 ± 25.1^a^	112.5 ± 20.4^a^	103.2 ± 17.5^a^	88.3 ± 12.4^a,b^

TG: triglycerides; TC: total cholesterol; HDL-C: high density lipoprotein cholesterol; ALT: alanine aminotransferase; AST: aspartate aminotransferase; BUN: blood urea nitrogen; SCr: serum creatinine; NC: normal control; DM: diabetes mellitus; DM + CL: diabetes with low-dose celastrol; DM + CM: diabetes with medium-dose celastrol; DM + CH: diabetes with high-dose celastrol. Data are expressed as mean ± SEM, ^a^ *P* < 0.05 versus NC group; ^b^ *P* < 0.05 versus DM group.
